# Dynamics of Tuberculosis (TB) with Drug Resistance to First-Line Treatment and Leaky Vaccination: A Deterministic Modelling Perspective

**DOI:** 10.1155/2021/5593864

**Published:** 2021-07-27

**Authors:** Dominic Otoo, Shaibu Osman, Stephen Atta Poku, Elvis Kobina Donkoh

**Affiliations:** ^1^Department of Mathematics and Statistics, University of Energy and Natural Resources, Sunyani, Ghana; ^2^Department of Basic Sciences, University of Health and Allied Sciences, Ho, Ghana

## Abstract

A deterministic model was formulated and employed in the analysis of the dynamics of tuberculosis with a keen emphasis on vaccination and drug resistance as the first line of treatment. It was assumed that some of the susceptible population were vaccinated but with temporal immunity. This is due to the fact that vaccines do not confer permanent immunity. Moreover, part of the infected individual after treatment grows resistance to the drug. Infective immigrants were also considered to be part of the population. The basic reproductive number for the model is estimated using the next-generation matrix method. The equilibrium points of the TB model and their local and global stability were determined. It was established that if the basic reproductive number was less than unity (*R*_0_ < 1), then the disease free equilibrium is stable and unstable if *R*_0_ > 1. Furthermore, we investigated the optimal prevention, treatment, and vaccination as control measures for the disease. As the objective functional was optimised, there have been a significant reduction in the number of infections and an increase in the number of recovery. The best control measure in combating tuberculosis infections is prevention and vaccination of the susceptible population.

## 1. Introduction

Respiratory disease can be described as an infection which can be treated with time. The commonest respiratory infections include pneumonia, tuberculosis, and flu. Chronic conditions such as asthma and chronic bronchitis are persistent and sometimes long-lasting [1].

Tuberculosis is among the most ancient diseases worldwide. It is very contagious. The causative organism, Mycobacterium tuberculosis, was discovered by the German microbiologist Robert Koch in 1882 [2]. The motivation behind this study is to use a deterministic model to analyse the dynamics of the infection and suggest the best optimal control measure in combating the disease.

Through coughing, singing, and sneezing, pulmonary tuberculosis is spread from a sick TB patient as a droplet infection. Inhalation by an uninfected individual of these droplets may cause infection. With the frequency and duration of contact with people who have the disease, the risk of contracting TB rises.

In 1993, the WHO decreed TB a global epidemic [3]. It is estimated that the risk of contracting active TB after coming into contact with an infected person is between 5% and 10%, with a greater proportion of the disease playing a crucial role which happens in the very first few years after the initial infection with the arrival of HIV [4].

Biological models usually explain the transmission dynamics of infectious diseases and can determine the status of the disease in a population with time. The basic reproduction number is the threshold value that determines the persistence of a disease in a population [5–7].

Optimal control theory is usually employed in biological models to determine the best optimal control strategy in combating infections in a population [8–10].

## 2. Model Description and Formulation

The model partitions the entire populace into six compartments according to their epidemiological status. We define *S*(*t*), *V*(*t*), *E*(*t*), *I*(*t*), *R*_1_(*t*), and *R*(*t*) as the number of susceptible individuals, vaccinated individuals, exposed individuals, infectious individuals, individuals with resistance to treatment, and recovered individuals, respectively, at time *t* ≥ 0.

Tables 1 and 2 show the variables and parameters used in the tuberculosis model.  Figure 1 shows the tuberculosis (TB) model transmission dynamics.

The following differential equations were obtained from the model flow diagram:

(1) $$\begin{array}{c} \frac{dS}{dt}=\Lambda +\alpha M+\sigma R-\beta SI-\left(\gamma +\mu \right)S, \end{array}$$

(2) $$\begin{array}{c} \frac{dV}{dt}\gamma S-\left(\theta +\mu \right)V, \end{array}$$

(3) $$\begin{array}{c} \frac{dE}{dt}=\beta SI-\left(\rho +\mu \right)E, \end{array}$$

(4) $$\begin{array}{c} \frac{dI}{dt}=\rho E+\left(1-\alpha \right)M-\left(\tau +\delta +\mu \right)I, \end{array}$$

(5) $$\begin{array}{c} \frac{dR_{1}}{dt}=\tau I-\left(\kappa +\mu \right)R_{1}, \end{array}$$

(6) $$\begin{array}{c} \frac{dR}{dt}=\kappa R_{1}+\theta V-\left(\sigma +\mu \right)R. \end{array}$$

Thus, the total population is given as

(7) $$\begin{array}{c} N=S+V+E+I+R_{1}+R, \end{array}$$

with initial conditions:

(8) $$\begin{array}{c} \left(S\left(0\right),V\left(0\right),E\left(0\right),I\left(0\right),R_{1}\left(0\right),R\left(0\right)\right)\in R_{+}^{6}. \end{array}$$

## 3. Tuberculosis Model Analysis

The tuberculosis (TB) model is about human population; hence, model state variables ought to be nonnegative and limited for all *t* ≥ 0. In this section, we demonstrate that the TB model is numerically and epidemiologically sensible.

### 3.1. Positivity of Solution

We prove the positivity of the variables in the model. Based on the concept of derivative of a function, the behavior of the function at a known point can be established.

**Theorem 1 .**

Let the initial set be *S*(0), *V*(0), *E*(0), *I*(0), *R*_1_(0), and *R*(0) and be nonnegative; then, the solution set of {*S*(*t*), *V*(*t*), *E*(*t*), *I*(*t*), *R*_1_(*t*), *R*(*t*)} of equation (1) is positive and bounded for all *t* > 0, wherever they exist.

**Proof**

From equation (1), we can state that

(9) $$\begin{array}{c} \frac{dS}{dt}\geq -\left(\gamma +\mu +\beta I\right)S,\\ \frac{dS}{S}\frac{dS}{dt}\geq -\left(\gamma +\mu +\beta I\right)dt,\\ \text{In }\left|S\right|\frac{dS}{dt}\geq -\left(\gamma +\mu +\beta I\right)t+c,\\ S\left(t\right)\frac{dS}{dt}\geq ce^{-\left(\gamma +\mu +\beta I\right)t}. \end{array}$$

At *t* = 0, *S*(0)(*dS*/*dt*) ≥ *c*,

(10) $$\begin{array}{c} S\left(t\right)\frac{dS}{dt}\geq S\left(0\right)e^{-\left(\gamma +\mu +\beta I\right)t}, \end{array}$$

since

(11) $$\begin{array}{c} \left(\gamma +\mu +\beta I\right)>0,S\left(t\right)\frac{dS}{dt}\geq 0. \end{array}$$

Also,

(12) $$\begin{array}{c} \frac{dV}{dt}\frac{dS}{dt}\geq -\left(\theta +\mu \right)V,\\ V\left(t\right)\frac{dS}{dt}\geq ce^{-\left(\theta +\mu \right)t}. \end{array}$$

At *t* = 0, *V*(0)(*dS*/*dt*) ≥ *c*,

(13) $$\begin{array}{c} V\left(t\right)\frac{dS}{dt}\geq V\left(0\right)e^{-\left(\theta +\mu \right)t}, \end{array}$$

since

(14) $$\begin{array}{c} \left(\theta +\mu \right)>0,V\left(t\right)\frac{dS}{dt}\geq 0. \end{array}$$

Also,

(15) $$\begin{array}{c} \frac{dE}{dt}\frac{dS}{dt}\geq -\left(\rho +\mu \right)E,\\ E\left(t\right)\frac{dS}{dt}\geq ce^{-\left(\rho +\mu \right)t}. \end{array}$$

At *t* = 0, *E*(0)(*dS*/*dt*) ≥ *c*,

(16) $$\begin{array}{c} E\left(t\right)\frac{dS}{dt}\geq E\left(0\right)e^{-\left(\rho +\mu \right)t}, \end{array}$$

since

(17) $$\begin{array}{c} \left(\rho +\mu \right)>0,E\left(t\right)\frac{dS}{dt}\geq 0. \end{array}$$

Also,

(18) $$\begin{array}{c} \frac{dI}{dt}\frac{dS}{dt}\geq -\left(\tau +\mu +\delta \right)I,\\ I\left(t\right)\frac{dS}{dt}\geq ce^{-\left(\tau +\mu +\delta \right)t}. \end{array}$$

At *t* = 0, *I*(0)(*dS*/*dt*) ≥ *c*,

(19) $$\begin{array}{c} I\left(t\right)\frac{dS}{dt}\geq I\left(0\right)e^{-\left(\tau +\mu +\delta \right)t}, \end{array}$$

since

(20) $$\begin{array}{c} \left(\tau +\mu +\delta \right)>0,I\left(t\right)\frac{dS}{dt}\geq 0. \end{array}$$

Also,

(21) $$\begin{array}{c} \frac{dR_{1}}{dt}\frac{dS}{dt}\geq -\left(\kappa +\mu \right)R_{1},\\ R_{1}\left(t\right)\frac{dS}{dt}\geq ce^{-\left(\kappa +\mu \right)t}. \end{array}$$

At *t* = 0, *R*_1_(0)(*dS*/*dt*) ≥ *c*,

(22) $$\begin{array}{c} R_{1}\left(t\right)\frac{dS}{dt}\geq R_{1}\left(0\right)e^{-\left(\kappa +\mu \right)t}, \end{array}$$

since

(23) $$\begin{array}{c} \left(\kappa +\mu \right)>0,R_{1}\left(t\right)\frac{dS}{dt}\geq 0. \end{array}$$

Also,

(24) $$\begin{array}{c} \frac{dR}{dt}\frac{dS}{dt}\geq -\left(\sigma +\mu \right)R,\\ R\left(t\right)\frac{dS}{dt}\geq ce^{-\left(\sigma +\mu \right)t}. \end{array}$$

At *t* = 0, *R*(0)(*dS*/*dt*) ≥ *c*,

(25) $$\begin{array}{c} R\left(t\right)\frac{dS}{dt}\geq R\left(0\right)e^{-\left(\sigma +\mu \right)t}, \end{array}$$

since

(26) $$\begin{array}{c} \left(\sigma +\mu \right)>0,R\left(t\right)\frac{dS}{dt}\geq 0. \end{array}$$

### 3.2. Boundedness of the System

The region in which solutions of the tuberculosis (TB) model system are uniformly bounded is the proper subset, and it is given by

(27) $$\begin{array}{c} \Gamma =\left\{\left(S,V,E,I,R_{1},R\right)\in R_{+}^{6}:N\leq \frac{\Lambda +M-\delta I}{\mu },\mu \neq 0\right\}. \end{array}$$

**Proof**

(28) $$\begin{array}{c} N=S+V+E+I+R_{1}+R,\\ \frac{dN}{dt}=\Lambda -\mu N+M-\delta I\frac{dN}{\Lambda -\mu N+M-\delta I}=dt-\frac{1}{\mu }\int \left(\frac{-\mu }{\Lambda -\mu N+M-\delta I}\right)dN=\int dt-\frac{1}{\mu }\text{In}\left|\Lambda -\mu N+M-\delta I\right|=t+c,\\ \text{In}\left|\Lambda -\mu N+M-dI\right|=-\mu t+c_{1},\\ \Lambda -\mu N+M-\delta I=c_{2}e^{-\mu t},\\ N\left(t\right)=\frac{\Lambda +M-\delta I-c_{2}e^{-\mu t}}{\mu },\\ \text{At }t=0,N\left(0\right)=N_{0},I\left(0\right)=I_{0},\\ N_{0}=\frac{\Lambda +M-\delta I_{0}-c_{2}}{\mu },\\ c_{2}=\Lambda +M-\delta I_{0}-\mu N_{0},\\ N\left(t\right)=\frac{\Lambda +M-\delta I-\left(\Lambda +M-\delta I_{0}-\mu N_{0}\right)e^{-\mu t}}{\mu }. \end{array}$$

So as *t*⟶∞, *N*⟶((*Λ* + *M* − *δI*)/*μ*) ∈ *R*_+_.

Therefore, Γ is a positive invariant.

### 3.3. Existence of Disease-Free Equilibrium Point

The disease-free equilibrium of the dynamical system (1) is obtained by setting *dS*/*dt* = *dV*/*dt* = *dE*/*dt* = *dI*/*dt* = *dR*_1_/*dt* = *dR*/*dt* = 0, and since there is no disease *E* = *I* = *R*_1_ = *R* = 0,

(29) $$\begin{array}{c} \Lambda +\alpha M-\left(\gamma +\mu \right)S=0\Rightarrow S=\frac{\Lambda +\alpha M}{\gamma +\mu }. \end{array}$$

Therefore, the disease-free equilibrium of the dynamical system (1) is

(30) $$\begin{array}{c} C^{0}=\left(S^{0},V^{0},E^{0},I^{0},R_{1}^{0},R^{0}\right)=\left(\frac{\Lambda +\alpha M}{\gamma +\mu },\frac{\gamma \left(\Lambda +\alpha M\right)}{\left(\theta +\mu \right)\left(\gamma +\mu \right)},0,0,0,0\right). \end{array}$$

### 3.4. Basic Reproductive Number

The basic reproductive number can be computed utilizing the cutting edge matrix approach. The basic reproduction number determines the state of a disease with time in a dynamical system [11, 12]. It is utilized to predict the stability of the disease equilibrium. The basic reproductive number is characterized as the quantity of secondary infections that one tainted person can create in a completely susceptible population [13, 14]. According to [13, 15], the next-generation matrix is defined as *K* = *FG*^−1^ and *R*_0_ = *ρ*(*FG*^−1^), where *ρ*(*FG*^−1^) denotes the spectral radius of *FG*^−1^.

Using the next-generation matrix, we consider only the infectious compartments in the system of differential equation in (1).

(31) $$\begin{array}{c} \frac{dE}{dt}=\beta SI-\left(\rho +\mu \right)E,\\ \frac{dI}{dt}=\rho E+\left(1-\alpha \right)M-\left(\tau +\delta +\mu \right)I,\\ \frac{dR_{1}}{dt}=\tau I-\left(\kappa +\mu \right)R_{1}. \end{array}$$

Let *f* be the count of emerging infection moving into the system and *g* be the count of infections exiting the system.

(32) $$\begin{array}{c} f=\left(\beta SI,0,0\right),\\ g=\left(\left(\rho +\mu \right)E,-\rho E-\left(1-\alpha \right)M+\left(\tau +\mu +\delta \right)I,-\gamma I+\left(k+\mu \right)R_{1}\right). \end{array}$$

The Jacobian matrix of *f* and *g* are obtained by

(33) $$\begin{array}{c} F=\left(\begin{array}{ccc} 0 & \beta S & 0\\ 0 & 0 & 0\\ 0 & 0 & 0 \end{array}\right),\\ G=\left(\begin{array}{ccc} \rho +\mu & 0 & 0\\ -\rho & \tau +\mu +\delta & 0\\ 0 & -\gamma & k+\mu \end{array}\right). \end{array}$$

But *R*_0_ = *ρ*(*FG*^−1^).

From the relation *FG*^−1^, the inverse of *G* can be calculated:

(34) $$\begin{array}{c} G^{-1}=\left(\begin{array}{ccc} \frac{\left(\gamma +\mu +\delta \right)}{\left(\rho +\mu \right)\left(\tau +\mu +\delta \right)} & 0 & 0\\ \frac{\rho }{\left(\rho +\mu \right)\left(\tau +\mu +\delta \right)} & \frac{1}{\left(\tau +\mu +\delta \right)} & 0\\ \frac{\gamma \rho }{\left(\rho +\mu \right)\left(\tau +\mu +\delta \right)\left(k+\mu \right)} & \frac{\gamma }{\left(\tau +\mu +\delta \right)\left(k+\mu \right)} & \frac{\left(\gamma +\mu +\delta \right)}{\left(\tau +\mu +\delta \right)\left(k+\mu \right)} \end{array}\right). \end{array}$$

Computing the product of *FG*^−1^,

(35) $$\begin{array}{c} FG^{-1}=\left(\begin{array}{ccc} 0 & \beta S & 0\\ 0 & 0 & 0\\ 0 & 0 & 0 \end{array}\right)\left(\begin{array}{ccc} \frac{\left(\gamma +\mu +\delta \right)}{\left(\rho +\mu \right)\left(\tau +\mu +\delta \right)} & 0 & 0\\ \frac{\rho }{\left(\rho +\mu \right)\left(\tau +\mu +\delta \right)} & \frac{1}{\left(\tau +\mu +\delta \right)} & 0\\ \frac{\gamma \rho }{\left(\rho +\mu \right)\left(\tau +\mu +\delta \right)\left(k+\mu \right)} & \frac{\gamma }{\left(\tau +\mu +\delta \right)\left(k+\mu \right)} & \frac{\left(\gamma +\mu +\delta \right)}{\left(\tau +\mu +\delta \right)\left(k+\mu \right)} \end{array}\right),\\ FG^{-1}=\left(\begin{array}{ccc} \frac{\beta \rho S}{\left(\rho +\mu \right)\left(\tau +\mu +\delta \right)} & \frac{\beta S}{\left(\tau +\mu +\delta \right)} & 0\\ 0 & 0 & 0\\ 0 & 0 & 0 \end{array}\right). \end{array}$$

By selecting the dominant eigenvalue of *FG*^−1^, the basic reproductive number is

(36) $$\begin{array}{c} R_{0}=\frac{\beta \rho S}{\left(\rho +\mu \right)\left(\tau +\mu +\delta \right)}. \end{array}$$

At the disease-free equilibrium, we substitute *S* = (*Λ* + *αM*)/(*γ* + *μ*) into the basic reproductive number, *R*_0_.

This therefore implies that

(37) $$\begin{array}{c} R_{0}=\frac{\beta \rho \left(\Lambda +\alpha M\right)}{\left(\gamma +\mu \right)\left(\rho +\mu \right)\left(\tau +\mu +\delta \right)}. \end{array}$$

### 3.5. Local Stability of the Disease-Free Equilibrium

**Theorem 2 .**

The disease-free equilibrium point *C*^0^ of the dynamical system (1) is locally asymptotically stable if *R*_0_ < 1 and unstable *R*_0_ > 1.

**Proof**

The Jacobian matrix of the dynamical system (1) at the DFE point *C*^0^ = ((*Λ* + *αM*)/(*γ* + *μ*), *γ*(*Λ* + *αM*)/(*θ* + *μ*)(*γ* + *μ*), 0, 0, 0, 0)

is given by

(38) $$\begin{array}{c} J\left(C^{0}\right)=\left(\begin{array}{cccccc} -\left(\gamma +\mu \right) & 0 & 0 & -\frac{\beta \left(\Lambda +\alpha M\right)}{\gamma +\mu } & 0 & \sigma \\ \gamma & -\left(\theta +\mu \right) & 0 & 0 & 0 & 0\\ 0 & 0 & -\left(\rho +\mu \right) & \frac{\beta \left(\Lambda +\alpha M\right)}{\gamma +\mu } & 0 & 0\\ 0 & 0 & \rho & -\left(\tau +\mu +\delta \right) & 0 & 0\\ 0 & 0 & 0 & \tau & -\left(\kappa +\mu \right) & 0\\ 0 & \theta & 0 & 0 & \kappa & -\left(\sigma +\mu \right) \end{array}\right). \end{array}$$

The corresponding characteristic equation for the eigenvalues *λ* is |*λI* − *J*(*C*^0^)| = 0.

(39) $$\begin{array}{c} \left|\begin{array}{cccccc} \lambda +\left(\gamma +\mu \right) & 0 & 0 & \frac{\beta \left(\Lambda +\alpha M\right)}{\gamma +\mu } & 0 & -\sigma \\ -\gamma & \lambda +\left(\theta +\mu \right) & 0 & 0 & 0 & 0\\ 0 & 0 & \lambda +\left(\rho +\mu \right) & -\frac{\beta \left(\Lambda +\alpha M\right)}{\gamma +\mu } & 0 & 0\\ 0 & 0 & -\rho & \lambda +\left(\tau +\mu +\delta \right) & 0 & 0\\ 0 & 0 & 0 & -\tau & \lambda +\left(\kappa +\mu \right) & 0\\ 0 & -\theta & 0 & 0 & -\kappa & \lambda +\left(\sigma +\mu \right) \end{array}\right|=0.\\ \begin{array}{c} \left(\lambda +\kappa +\mu \right)\left[\left(\lambda +\gamma +\mu \right)\left(\lambda +\theta +\mu \right)\left(\lambda +\sigma +\mu \right)-\gamma \theta \sigma \right]\\ \left[\left(\lambda +\tau +\mu +\delta \right)\left(\lambda +\rho +\mu \right)-\frac{\rho \beta \left(\Lambda +\alpha M\right)}{\gamma +\mu }\right]=0, \end{array}\\ \lambda +\kappa +\mu =0\Rightarrow \lambda_{1}=-\kappa -\mu ,\\ \left(\lambda +\gamma +\mu \right)\left(\lambda +\theta +\mu \right)\left(\lambda +\sigma +\mu \right)-\sigma \gamma \theta =0,\\ \lambda^{3}+\left(\gamma +\theta +\sigma +3\mu \right)\lambda^{2}+\left[\left(\theta +\mu \right)\left(\sigma +\mu \right)\left(\gamma +\mu \right)\left(\theta +\sigma +2\mu \right)\right]\lambda +\left[\mu^{3}+\left(\gamma +\theta +\sigma \right)\mu^{2}+\left(\gamma \theta +\sigma \gamma +\sigma \theta \right)\mu \right]=0. \end{array}$$

This is

(40) $$\begin{array}{c} \lambda^{3}+Q\lambda^{2}+R\lambda +T=0. \end{array}$$

According to the Routh-Hurwitz criterion, since *Q* > 0, *R* > 0, and *T* > 0, *λ*_2_, *λ*_3_, and *λ*_4_ will have negative real part as roots.

Also,

(41) $$\begin{array}{c} \left(\rho +\mu \right)\left(\tau +\mu +\delta \right)-\frac{\rho \beta \left(\Lambda +\alpha M\right)}{\gamma +\mu }>0,\\ \lambda^{2}+\left(\rho +\tau +\delta +2\mu \right)\lambda +\left(\rho +\mu \right)\left(\tau +\mu +\delta \right)-\frac{\rho \beta \left(\Lambda +\alpha M\right)}{\gamma +\mu }=0. \end{array}$$

The roots, *λ*_5_ and *λ*_6_, of this characteristic polynomial will have negative real part if and only if

(42) $$\begin{array}{c} \left(\rho +\mu \right)\left(\tau +\mu +\delta \right)-\frac{\rho \beta \left(\Lambda +\alpha M\right)}{\gamma +\mu }>0,\\ 1-\frac{\rho \beta \left(\Lambda +\alpha M\right)}{\left(\gamma +\mu \right)\left(\rho +\mu \right)\left(\tau +\mu +\delta \right)}>0,\\ 1-R_{0}>0,\\ R_{0}<1. \end{array}$$

Therefore, *C*^0^ is asymptotically stable since *R*_0_ < 1 and unstable if *R*_0_ > 1.

### 3.6. Global Stability of the Disease-Free Equilibrium

**Theorem 3 .**

The disease-free equilibrium point *C*^0^ of the dynamical system (1) is globally asymptotically stable in *Λ* if *R*_0_ < 1 and unstable *R*_0_ > 1.

**Proof**

Using the Perron eigenvector to prove the global stability of the disease free equilibrium as in [16–18], we apply the matrix-theoretic method. In the dynamical system, the disease compartment is $x={\left(\begin{array}{ccc} E & I & R_{1} \end{array}\right)}^{T}\in R^{3}$ and the nondisease compartment is *y* ∈ *R*^6^.

Taking the same path as [16, 18], let us set

(43) $$\begin{array}{c} f\left(x,y\right)≔\left(F-G\right)x-F\left(x,y\right)+G\left(x,y\right). \end{array}$$

Then, the equation of the disease compartment can be written as

(44) $$\begin{array}{c} x^{1}=\left(F-G\right)x-f\left(x,y\right). \end{array}$$

**Theorem 4 .**

Let *R*_*o*_ be defined as in equation (11). Then, the threshold property holds for system (1).

**Proof**

Using the condition outlined in Theorem 3, we set the Lyapunov function for the disease-free equilibrium (DFE).

We first find *w*^*T*^ (the left eigenvector of the nonnegative matrix *G*^−1^*F*):

(45) $$\begin{array}{c} G^{-1}F=\left(\begin{array}{ccc} \frac{1}{\left(\rho +\mu \right)} & 0 & 0\\ \frac{\rho }{\left(\rho +\mu \right)\left(\gamma +\mu +\delta \right)} & \frac{1}{\left(\gamma +\mu +\delta \right)} & 0\\ \frac{\gamma \rho }{\left(\rho +\mu \right)\left(\gamma +\mu +\delta \right)\left(\kappa +\mu \right)} & \frac{\gamma }{\left(\gamma +\mu +\delta \right)\left(\kappa +\mu \right)} & \frac{1}{\left(\kappa +\mu \right)} \end{array}\right)\left(\begin{array}{ccc} 0 & \beta S & 0\\ 0 & 0 & 0\\ 0 & 0 & 0 \end{array}\right)=\left(\begin{array}{ccc} 0 & \frac{\beta S}{\left(\rho +\mu \right)} & 0\\ 0 & \frac{\rho \beta S}{\left(\rho +\mu \right)\left(\gamma +\mu +\delta \right)} & 0\\ 0 & \frac{\rho \beta \gamma S}{\left(\rho +\mu \right)\left(\gamma +\mu +\delta \right)\left(\kappa +\mu \right)} & 0 \end{array}\right)=\left(\begin{array}{ccc} 0 & R_{0}\frac{\left(\gamma +\mu +\delta \right)}{\rho } & 0\\ 0 & R_{0} & 0\\ 0 & R_{0}\frac{\gamma }{\kappa +\mu } & 0 \end{array}\right)\Rightarrow w^{T}=\left(\begin{array}{ccc} 0 & R_{0}\frac{\left(\gamma +\mu +\delta \right)}{\rho } & 0\\ 0 & R_{0} & 0\\ 0 & R_{0}\frac{\gamma }{\kappa +\mu } & 0 \end{array}\right)\left(\begin{array}{c} n_{1}\\ n_{2}\\ n_{3} \end{array}\right)=\left(\begin{array}{c} n_{1}\\ n_{2}\\ n_{3} \end{array}\right)R_{0}\Rightarrow R_{0}\frac{\left(\gamma +\mu +\delta \right)}{\rho }n_{2}=R_{0}n_{1},R_{0}n_{2}=R_{0}n_{2}\text{ and }R_{0}\frac{\gamma }{\kappa +\mu }n_{2}=R_{0}n_{3}. \end{array}$$

$∴w^{T}=\left(\begin{array}{ccc} \left(\gamma +\mu +\delta \right)/\rho & 1 & \gamma /\left(\kappa +\mu \right) \end{array}\right)$, and any multiple of this becomes our eigenvector.

From equation (40),

(46) $$\begin{array}{c} x^{1}=\left(F-G\right)x-f\left(x,y\right). \end{array}$$

That is, *f*(*x*, *y*) = (*F* − *G*)*x* − *x*^1^,

(47) $$\begin{array}{c} f\left(x,y\right)=\left[\left(\begin{array}{ccc} 0 & \beta S & 0\\ 0 & 0 & 0\\ 0 & 0 & 0 \end{array}\right)-\left(\begin{array}{ccc} \rho +\mu & 0 & 0\\ -\rho & \tau +\mu +\delta & 0\\ 0 & -\gamma & \kappa +\mu \end{array}\right)\right]x-\left(\begin{array}{c} \beta SI\\ 0\\ 0 \end{array}\right)+\left(\begin{array}{c} \left(\rho +\mu \right)E\\ -\rho E+\left(1-\alpha \right)M+\left(\tau +\mu +\delta \right)I\\ -\gamma I+\left(\kappa +\mu \right)R_{1} \end{array}\right)=\left(\begin{array}{ccc} -\left(\rho +\mu \right) & \beta S & 0\\ \rho & -\left(\tau +\mu +\delta \right) & 0\\ 0 & \gamma & -\left(\kappa +\mu \right) \end{array}\right)\left(\begin{array}{c} E\\ I\\ R_{1} \end{array}\right)+\left(\begin{array}{c} -\beta SI+\left(\rho +\mu \right)E\\ -\rho E+\left(1-\alpha \right)M+\left(\tau +\mu +\delta \right)I\\ -\gamma I+\left(\kappa +\mu \right)R_{1} \end{array}\right)=\left(\begin{array}{c} \beta SI-\left(\rho +\mu \right)E\\ \rho E-\left(\tau +\mu +\delta \right)I\\ \gamma I-\left(\kappa +\mu \right)R_{1} \end{array}\right)+\left(\begin{array}{c} -\beta SI+\left(\rho +\mu \right)E\\ -\rho E+\left(1-\alpha \right)M+\left(\tau +\mu +\delta \right)I\\ -\gamma I+\left(\kappa +\mu \right)R_{1} \end{array}\right)=0, \end{array}$$

where *α* = 1 at the disease-free equilibrium.

Therefore, *f*(*x*, *y*) = 0, and this satisfies the demand of Theorem 4. The Lyapunov function *D* is

(48) $$\begin{array}{c} D=w^{T}G^{-1}x,\\ D=\left(\begin{array}{ccc} \frac{\gamma +\mu +\delta }{\rho } & 1 & \frac{\gamma }{\kappa +\mu } \end{array}\right)\left(\begin{array}{ccc} \frac{1}{\left(\rho +\mu \right)} & 0 & 0\\ \frac{\rho }{\left(\rho +\mu \right)\left(\gamma +\mu +\delta \right)} & \frac{1}{\left(\gamma +\mu +\delta \right)} & 0\\ \frac{\rho \gamma }{\left(\rho +\mu \right)\left(\gamma +\mu +\delta \right)\left(\kappa +\mu \right)} & \frac{\gamma }{\left(\gamma +\mu +\delta \right)\left(\kappa +\mu \right)} & \frac{1}{\left(\kappa +\mu \right)} \end{array}\right)\left(\begin{array}{c} E\\ I\\ R_{1} \end{array}\right)=\left(\begin{array}{ccc} \frac{\gamma +\mu +\delta }{\rho } & 1 & \frac{\gamma }{\kappa +\mu } \end{array}\right)\left(\begin{array}{c} \frac{1}{\left(\rho +\mu \right)}E\\ \frac{\rho }{\left(\rho +\mu \right)\left(\gamma +\mu +\delta \right)}E+\frac{1}{\left(\gamma +\mu +\delta \right)}I\\ \frac{\rho \gamma }{\left(\rho +\mu \right)\left(\gamma +\mu +\delta \right)\left(\kappa +\mu \right)}E+\frac{\gamma }{\left(\gamma +\mu +\delta \right)\left(\kappa +\mu \right)}I+\frac{1}{\left(\kappa +\mu \right)}R_{1} \end{array}\right)=\left(\left(\frac{\gamma +\mu +\delta }{\rho \left(\rho +\mu \right)}+\frac{\rho }{\left(\rho +\mu \right)\left(\gamma +\mu +\delta \right)}+\frac{\rho \gamma^{2}}{\left(\rho +\mu \right)\left(\gamma +\mu +\delta \right){\left(\kappa +\mu \right)}^{2}}\right)E+\left(\frac{1}{\left(\gamma +\mu +\delta \right)}+\frac{\gamma^{2}}{\left(\gamma +\mu +\delta \right){\left(\kappa +\mu \right)}^{2}}\right)I+\frac{\gamma }{{\left(\kappa +\mu \right)}^{2}}R_{1}\right)=\left(\frac{{\left(\gamma +\mu +\delta \right)}^{2}{\left(\kappa +\mu \right)}^{2}+\rho^{2}\left(\rho +\mu \right)\left(\kappa +\mu \right)+\rho^{2}\gamma^{2}}{\rho \left(\rho +\mu \right)\left(\gamma +\mu +\delta \right){\left(\kappa +\mu \right)}^{2}}\right)E+\left(\frac{{\left(\kappa +\mu \right)}^{2}+\gamma^{2}}{\left(\gamma +\mu +\delta \right){\left(\kappa +\mu \right)}^{2}}\right)I+\left(\frac{\gamma }{{\left(\kappa +\mu \right)}^{2}}\right)R_{1}. \end{array}$$

But

(49) $$\begin{array}{c} D^{1}=w^{T}V^{-1}x^{1}=w^{T}V^{-1}\left(F-V\right)x-w^{T}V^{-1}f\left(x,y\right),\\ D^{1}=\left(R_{0}-1\right)w^{T}x-w^{T}V^{-1}f\left(x,y\right). \end{array}$$

Since *w*^*T*^ > 0, *V*^−1^, and *f*(*x*, *y*) = 0,

(50) $$\begin{array}{c} \Rightarrow D^{1}<0\text{ if }R_{0}<1. \end{array}$$

From the derivative of the Lyapunov function, *D*^1^ < 0 when *R*_0_ < 1, which satisfies the condition that the disease-free equilibrium is asymptotically stable and unstable when *R*_0_ > 1.

### 3.7. Existence of the Endemic Equilibrium

The endemic equilibrium point is acquired by mounting the right-hand side of the dynamical system (1) equal to zero and solving them simultaneously [19, 20]. The endemic equilibrium point is *C*^∗^ = (*S*^∗^, *V*^∗^, *E*^∗^, *I*^∗^, *R*_1_^∗^, *R*^∗^), where

(51) $$\begin{array}{c} S^{*}=\frac{\left(\theta +\mu \right)\left[\left(\Lambda +\alpha M\right)\left(\sigma +\mu \right)\left(\kappa +\mu \right)+\kappa \sigma \tau I^{*}\right]}{\left(\kappa +\mu \right)\left[\left(\sigma +\mu \right)\left(\theta +\mu \right)\left(\gamma +\mu +\beta I^{*}\right)-\sigma \theta \gamma \right]},\\ V^{*}=\frac{\gamma \left[\left(\Lambda +\alpha M\right)\left(\sigma +\mu \right)\left(\kappa +\mu \right)+\kappa \sigma \tau I^{*}\right]}{\left(\kappa +\mu \right)\left[\left(\sigma +\mu \right)\left(\theta +\mu \right)\left(\gamma +\mu +\beta I^{*}\right)-\sigma \theta \gamma \right]},\\ E^{*}=\frac{\beta \left(\theta +\mu \right)\left[\left(\Lambda +\alpha M\right)\left(\sigma +\mu \right)\left(\kappa +\mu \right)+\kappa \sigma \tau I^{*}\right]I^{*}}{\left(\rho +\mu \right)\left(\kappa +\mu \right)\left[\left(\sigma +\mu \right)\left(\theta +\mu \right)\left(\gamma +\mu +\beta I^{*}\right)-\sigma \theta \gamma \right]},\\ R_{1}^{*}=\frac{\tau I^{*}}{\left(\kappa +\mu \right)},\\ R^{*}=\frac{1}{\left(\sigma +\mu \right)\left(\kappa +\mu \right)}\left[\kappa \tau I^{*}+\frac{\theta \gamma \left[\left(\Lambda +\alpha M\right)\left(\sigma +\mu \right)\left(\kappa +\mu \right)+\kappa \sigma \tau I^{*}\right]}{\left[\left(\sigma +\mu \right)\left(\theta +\mu \right)\left(\gamma +\mu +\beta I^{*}\right)-\sigma \theta \gamma \right]}\right]. \end{array}$$

*I* ^∗^ is the positive root of *AI*^∗^^2^ + *BI*^∗^ + *C* = 0, that is, $I^{*}=-\left(B+\sqrt{B^{2}-4AC}\right)/2A>0$.

We have three possibilities of getting the value of *I*^∗^:

1. If *B*^2^ − 4*AC* < 0, then there is no endemic equilibrium state
2. If *B*^2^ − 4*AC* = 0, then again, the endemic equilibrium point does not exist
3. If *B*^2^ − 4*AC* > 0, then the endemic equilibrium point exists when *AC* < 0

where *A* = *κστρβ*(*θ* + *μ*),

(52) $$\begin{array}{c} B=\beta \left(\sigma +\mu \right)\left(\kappa +\mu \right)\left[\rho \left(\theta +\mu \right)\left(\Lambda +\alpha M\right)+\left(\rho +\mu \right)\left(\tau +\mu +\delta \right)\left(\theta +\mu \right)+\left(\rho +\mu \right)\left(1-\alpha \right)M\right],\\ C=\left(\rho +\mu \right)\left(\kappa +\mu \right)\left[\theta \gamma \sigma -\left(\sigma +\mu \right)\left(\theta +\mu \right)\left(\gamma +\mu \right)\right]\left[\left(\tau +\mu +\delta \right)-\left(1-\alpha \right)M\right]. \end{array}$$

### 3.8. Local Stability of the Endemic Equilibrium

**Theorem 5 .**

The positive endemic equilibrium point *C*^∗^ of the system (1) is locally asymptotically stable if *R*_*o*_ > 1.

**Proof**

The Jacobian matrix of the system of equation (1) at the endemic point is

(53) $$\begin{array}{c} J\left(C^{*}\right)=\left(\begin{array}{cccccc} M_{11} & 0 & 0 & M_{14} & 0 & \sigma \\ \gamma & M_{22} & 0 & 0 & 0 & 0\\ M_{31} & 0 & M_{33} & M_{34} & 0 & 0\\ 0 & 0 & \rho & M_{44} & 0 & 0\\ 0 & 0 & 0 & \tau & M_{55} & 0\\ 0 & \theta & 0 & 0 & \kappa & M_{66} \end{array}\right), \end{array}$$

where *M*_11_ = −(*γ* + *μ* + *βI*^∗^), *M*_14_ = −*βS*^∗^, *M*_22_ = −(*θ* + *μ*), *M*_31_ = −*βI*^∗^, *M*_33_ = −(*ρ* + *μ*), *M*_34_ = −*βS*^∗^, *M*_44_ = −(*τ* + *μ* + *δ*), *M*_55_ = −(*κ* + *μ*), and *M*_66_ = −(*σ* + *μ*).

The corresponding characteristic equation is *J*(*C*^∗^) denoted by |*λI* − *J*(*C*^∗^)| = 0 and is given as

(54) $$\begin{array}{c} \left|\begin{array}{cccccc} \lambda -M_{11} & 0 & 0 & M_{14} & 0 & \sigma \\ \gamma & \lambda -M_{22} & 0 & 0 & 0 & 0\\ M_{31} & 0 & \lambda -M_{33} & M_{34} & 0 & 0\\ 0 & 0 & \rho & \lambda -M_{44} & 0 & 0\\ 0 & 0 & 0 & \tau & \lambda -M_{55} & 0\\ 0 & \theta & 0 & 0 & \kappa & \lambda -M_{66} \end{array}\right|=0. \end{array}$$

The matrix *J*(*C*^∗^) is a strictly column diagonally dominant matrix. Again, all the diagonal entries are negative. Hence, all eigenvalues of *J*(*C*^∗^) have negative real part. Now applying the Gershgorin circle theorem [21], *C*^∗^ is locally asymptotically stable if |*M*_11_| > |*M*_14_ + *σ*|, |*M*_22_| > |*γ*|, |*M*_33_| > |*M*_31_ + *M*_34_|, |*M*_44_| > |*ρ*|, |*M*_55_| > |*τ*|, and |*M*_66_| > |*θ* + *κ*|.

### 3.9. Global Stability of the Endemic Equilibrium

**Theorem 6 .**

The dynamical system (1) is said to have an endemic equilibrium if *R*_*o*_ > 1, and it is globally asymptotically stable.

**Proof**

Consider the Lyapunov function defined by

(55) $$\begin{array}{c} Q\left(C^{*}\right)=\left(S-S^{*}-S^{*}\text{In}\frac{S^{*}}{S}\right)+\left(V-V^{*}-V^{*}\text{In}\frac{V^{*}}{V}\right)+\left(E-E^{*}-E^{*}\text{In}\frac{E^{*}}{E}\right)+\left(I-I^{*}-I^{*}\text{In}\frac{I^{*}}{I}\right)+\left(R_{1}-R_{1}^{*}-R_{1}^{*}\text{In}\frac{R_{1}^{*}}{R_{1}}\right)+\left(R-R^{*}-R^{*}\text{In}\frac{R^{*}}{R}\right). \end{array}$$

Computing the derivative of *Q* along the solution of the dynamical system in (1) directly,

(56) $$\begin{array}{c} \frac{dQ}{dt}=\left(\frac{S-S^{*}}{S}\right)\frac{dS}{dt}+\left(\frac{V-V^{*}}{V}\right)\frac{dV}{dt}+\left(\frac{E-E^{*}}{E}\right)\frac{dE}{dt}+\left(\frac{I-I^{*}}{I}\right)\frac{dI}{dt}+\left(\frac{R_{1}-R_{1}^{*}}{R_{1}}\right)\frac{dR_{1}}{dt}+\left(\frac{R-R^{*}}{R}\right)\frac{dR}{dt},\\ \frac{dQ\left(C^{*}\right)}{dt}=\left(\frac{S-S^{*}}{S}\right)\left(\Lambda +\alpha M+\sigma R-\left(\gamma +\mu \right)S-\beta SI\right)+\left(\frac{V-V^{*}}{V}\right)\left(\gamma S-\left(\theta +\mu \right)S\right)+\left(\frac{E-E^{*}}{E}\right)\left(\beta SI-\left(\rho +\mu \right)E\right)+\left(\frac{I-I^{*}}{I}\right)\left(\rho E+\left(1-\alpha \right)M-\left(\tau +\delta +\mu \right)I\right)+\left(\frac{R_{1}-R_{1}^{*}}{R_{1}}\right)\left(\tau I-\left(\kappa +\mu \right)R_{1}\right)+\left(\frac{R-R^{*}}{R}\right)\left(\kappa R_{1}+\theta V-\left(\sigma +\mu \right)R\right),\\ \frac{dQ}{dt}=\left(\Lambda +M+\mu N^{*}+\gamma S^{*}+\sigma V^{*}+\rho E^{*}+\left(\tau +\delta \right)I^{*}+\kappa R_{1}^{*}+\sigma R^{*}+\beta S^{*}I\right)-\left(\mu N+\left(\Lambda +\alpha M+\sigma R\right)\frac{S^{*}}{S}+\gamma \frac{SV^{*}}{V}+\beta \frac{SIE^{*}}{E}+\delta I+\left(\rho E+\left(1-\alpha \right)M\right)\frac{I^{*}}{I}+\tau \frac{IR_{1}^{*}}{R_{1}}+\left(\kappa R_{1}+\theta V\right)\frac{R^{*}}{R}\right)\Rightarrow \frac{dQ}{dt}=Z-Y, \end{array}$$

where *Z* = *Λ* + *M* + *μN*^∗^ + *γS*^∗^ + *σV*^∗^ + *ρE*^∗^ + (*τ* + *δ*)*I*^∗^ + *κR*_1_^∗^ + *σR*^∗^ + *βS*^∗^*I* and *Y* = *μN* + (*Λ* + *αM* + *σR*)(*S*^∗^/*S*) + *γ*(*SV*^∗^/*V*) + *β*(*SIE*^∗^/*E*) + *δI* + (*ρE* + (1 − *α*)*M*)(*I*^∗^/*I*) + *τ*(*IR*_1_^∗^/*R*_1_) + (*κR*_1_ + *θV*)(*R*^∗^/*R*).

Imposing the condition that *Z* < *Y*, the derivative of the Lyapunov function with respect to time is less than or equal to zero.

If *Z* < *Y*, then *dQ*/*dt* ≤ 0.

But *dQ*/*dt* = 0 if and only if *S* = *S*^∗^, *V* = *V*^∗^, *E* = *E*^∗^, *I* = *I*^∗^, *R*_1_ = *R*_1_^∗^, and *R* = *R*^∗^.

Therefore, the endemic equilibrium point *C*^∗^ is globally asymptotically stable in Γ if *Z* < *Y*.

The largest invariant set in {*C*^∗^ = (*S*^∗^, *V*^∗^, *E*^∗^, *I*^∗^, *R*_1_^∗^, *R*^∗^) ∈ Γ : *dQ*/*dt* = 0} is a singleton, where *C*^∗^ is the endemic equilibrium point.

## 4. TB Model Extension to Optimal Control

An analysis of the optimal controls to ascertain its effects on the model is been conducted. The optimal control problem is obtained by integrating the undermentioned control functions into the tuberculosis model (1) and introducing an objective functional that desires to minimize the controls (*u*_1_, *u*_2_, *u*_3_), where *u*_1_ is the vaccination of the susceptible population (*S*) as a control measure, *u*_2_ is the treatment of the infected individuals (*I*) as a control measure, and *u*_3_ is the education/sensitization of the exposed population (*E*) as a control measure.

By inserting the various controls, the system with the optimal controls becomes

(57) $$\begin{array}{c} \frac{dS}{dt}=\Lambda +\alpha M+\sigma R-u_{1}\gamma S-\mu S-\beta SI, \end{array}$$

(58) $$\begin{array}{c} \frac{dV}{dt}=u_{1}\gamma S-\left(\theta +\mu \right)V, \end{array}$$

(59) $$\begin{array}{c} \frac{dE}{dt}=\beta SI-\left(1-u_{3}\right)\rho E-\mu E, \end{array}$$

(60) $$\begin{array}{c} \frac{dI}{dt}=\left(1-u_{3}\right)\rho E+\left(1-\alpha \right)M-u_{2}\tau I-\left(\delta +\mu \right)I, \end{array}$$

(61) $$\begin{array}{c} \frac{dR_{1}}{dt}u_{2}\tau I-\left(1-u_{2}\right)\kappa R_{1}-\mu R_{1}, \end{array}$$

(62) $$\begin{array}{c} \frac{dR}{dt}\left(1-u_{2}\right)\kappa R_{1}-\left(1-u_{1}\right)\theta V-\left(\sigma +\mu \right)R. \end{array}$$

Let the optimal levels of the control set be *u*, which is Lebesgue measurable and defined as

(63) $$\begin{array}{c} U=\left\{\left(u_{1}\left(t\right),u_{2}\left(t\right),u_{3}\left(t\right)\right)\text{: }0\leq u_{1}<1,0\leq u_{2}<1,0\leq u_{3}<1,0\leq t\leq t_{f}\right\}. \end{array}$$

The quadratic nature of the control efforts as a result of the assumption that costs is generally nonlinear in nature. Our objective is to minimise the number of infections and reduce the cost of treatment.

The problem is to find a control *u*(*t*) and its associated state variables *S*(*t*), *V*(*t*), *E*(*t*), *I*(*t*), *R*_1_(*t*), and *R*(*t*) to minimize the objective functional *J* given by

(64) $$\begin{array}{c} J=\underset{\left(u_{1},u_{2},u_{3}\right)}{\min}\int_{0}^{t_{f}}\left(a_{1}I+a_{2}R_{1}+\overset{3}{\underset{i=1}{\sum }}w_{i}{u_{i}}^{2}\right)dt. \end{array}$$

That is, *J* = min_(*u*_1_, *u*_2_, *u*_3_)_∫_0_^*t*_*f*_^(*a*_1_*I* + *a*_2_*R*_1_ + *w*_1_*u*_1_^2^ + *w*_2_*u*_2_^2^ + *w*_3_*u*_3_^2^)*dt* subject to the differential equation system (57), where *a*_1_, *a*_2_, *w*_1_, *w*_2_, and *w*_3_ are the weight constants to balance the terms in the integrals to abstain the ascendance of one over the others.

Also, *a*_1_, *I*, and *a*_2_*R*_1_ are the cost associated with the infected individuals and the individuals with resistance to treatment, respectively, while *w*_1_*u*_1_^2^, *w*_2_*u*_2_^2^, and *w*_3_*u*_3_^2^ are the cost associated with vaccination, treatment, and sensitization as preventive measures. *t*_*f*_ is the period of the intervention.

The purpose of inserting the controls is to minimize the number of infections and at the same time reduce the cost of treatment.

Our task at this point is to find the optimal functions: *u*_1_^∗^(*t*), *u*_2_^∗^(*t*), and *u*_3_^∗^(*t*) such that *J*(*u*_1_^∗^(*t*), *u*_1_^∗^(*t*), *u*_1_^∗^(*t*)) = min_(*u*_1_, *u*_2_, *u*_3_)_ ∈ ∪*J*(*u*_1_, *u*_2_, *u*_3_), where *U* = {*u*_*i*_ : 0 ≤ *u*_*i*_(*t*) ≤ 1, *t* ∈ [0, *t*_*f*_], *i* = 1, 2, 3} is referred to as the control set.

### 4.1. Pontryagin's Maximum Principle

Consider the Lagrangian function:

(65) $$\begin{array}{c} L\left(I,R_{1},u_{1},u_{2},u_{3},t\right)=a_{1}I+a_{2}R_{1}+w_{1}u_{1}^{2}+w_{2}u_{2}^{2}+w_{3}u_{3}^{2}. \end{array}$$

The Pontryagin maximum principle provides the essential condition that the optimal must satisfy. This changes the system of the differential equation into minimization problem pointwise Hamiltonian (*H*) with respect to (*u*_1_, *u*_2_, *u*_3_).

Hence, the Hamiltonian (*H*) becomes

(66) $$\begin{array}{c} H\left(S,V,E,I,R_{1},R,t\right)=L\left(I,R_{1},u_{1},u_{2},u_{3},t\right)+\lambda_{1}\frac{dS}{dt}+\lambda_{2}\frac{dV}{dt}+\lambda_{3}\frac{dE}{dt}+\lambda_{4}\frac{dI}{dt}+\lambda_{5}\frac{dR_{1}}{dt}+\lambda_{6}\frac{dR}{dt}, \end{array}$$

where *λ*_1_, *λ*_2_, *λ*_3_, *λ*_4_, *λ*_5_, and *λ*_6_ are disjoint variables.

(67) $$\begin{array}{c} H=a_{1}I+a_{2}R_{1}+w_{1}u_{1}^{2}+w_{2}u_{2}^{2}+w_{3}u_{3}^{2}+\lambda_{1}\left\{\Lambda +\alpha M+\sigma R-u_{1}\gamma S-\mu S-\beta SI\right\}+\lambda_{2}\left\{u_{1}\gamma S-\left(\theta +\mu \right)V\right\}+\lambda_{3}\left\{\beta SI-\left(1-u_{3}\right)\rho E-\mu E\right\}+\lambda_{4}\left\{\left(1-u_{3}\right)\rho E+\left(1-\alpha \right)M-u_{2}\tau I-\left(\delta +\mu \right)I\right\}+\lambda_{5}\left\{u_{2}\tau I-\left(1-u_{2}\right)\kappa R_{1}-\mu R_{1}\right\}+\lambda_{6}\left\{\left(1-u_{2}\right)\kappa R_{1}+\left(1-u_{1}\right)\theta V-\left(\sigma +\mu \right)R\right\}, \end{array}$$

considering the relation

(68) $$\begin{array}{c} \frac{d\lambda_{i}}{dt}=-\frac{\partial H}{\partial \overset{•}{x}\left(t\right)}. \end{array}$$

By taking partial derivatives of the Hamiltonian function with respect to (*S*, *V*, *E*, *I*, *R*_1_, *R*) and negating each of them, the following costate variables are the solutions of the adjoint systems.

(69) $$\begin{array}{c} \frac{d\lambda_{1}}{dt}=-\frac{\partial H}{\partial S}=\left(\lambda_{1}-\lambda_{2}\right)u_{1}\gamma +\left(\lambda_{1}-\lambda_{3}\right)\beta I+\mu \lambda_{1},\\ \frac{d\lambda_{2}}{dt}=-\frac{\partial H}{\partial V}=\left(\lambda_{2}-\lambda_{6}\right)\theta +u_{2}\lambda_{2}+u_{1}\theta \lambda_{6},\\ \frac{d\lambda_{3}}{dt}-\frac{\partial H}{\partial E}=\left(1-u_{3}\right)\left(\lambda_{3}-\lambda_{4}\right)\rho +\mu \lambda_{3},\\ \frac{d\lambda_{4}}{dt}-\frac{\partial H}{\partial I}=\left(\lambda_{1}-\lambda_{3}\right)\beta S+\left(\lambda_{4}-\lambda_{5}\right)u_{2}\tau +\left(\mu +\delta \right)\lambda_{4},\\ \frac{d\lambda_{5}}{dt}-\frac{\partial H}{\partial R_{1}}=\left(1-u_{2}\right)\left(\lambda_{5}-\lambda_{6}\right)\kappa +\mu \lambda_{5},\\ \frac{d\lambda_{6}}{dt}-\frac{\partial H}{\partial R}=\left(\lambda_{6}-\lambda_{1}\right)\sigma +\mu \lambda_{6}. \end{array}$$

The above satisfy the transversality condition:

(70) $$\begin{array}{c} \lambda_{1}\left(t_{f}\right)=\lambda_{2}\left(t_{f}\right)=\lambda_{3}\left(t_{f}\right)=\lambda_{4}\left(t_{f}\right)=\lambda_{5}\left(t_{f}\right)=\lambda_{6}\left(t_{f}\right)=0. \end{array}$$

Moreover, the characterization of the optimal control is obtained by solving

(71) $$\begin{array}{c} \frac{\partial H}{\partial u_{i}}=0, \end{array}$$

where *u*_*i*_ = *u*_*i*_^∗^, *i* = 1, 2, 3.

(72) $$\begin{array}{c} \frac{\partial H}{\partial u_{1}}=2w_{1}u_{1}+\left(\lambda_{2}-\lambda_{1}\right)\gamma S-\lambda_{6}\theta V\Rightarrow 2w_{1}u_{1}+\left(\lambda_{2}-\lambda_{1}\right)\gamma S-\lambda_{6}\theta V=0∴u_{1}^{*}=\frac{\left(\lambda_{1}-\lambda_{2}\right)\gamma S^{*}+\lambda_{6}\theta V^{*}}{2w_{1}},\\ \frac{\partial H}{\partial u_{2}}=2w_{2}u_{2}-\left(\lambda_{4}-\lambda_{5}\right)\tau I^{*}-\left(\lambda_{6}-\lambda_{5}\right)\kappa R_{1}^{*}\Rightarrow 2w_{2}u_{2}-\left(\lambda_{4}-\lambda_{5}\right)\tau I^{*}-\left(\lambda_{6}-\lambda_{5}\right)\kappa R_{1}^{*}=0∴u_{2}^{*}=\frac{\left(\lambda_{4}-\lambda_{5}\right)\tau I^{*}+\left(\lambda_{6}-\lambda_{5}\right)\kappa R_{1}^{*}}{2w_{2}},\\ \frac{\partial H}{\partial u_{3}}=2w_{3}u_{3}-\left(\lambda_{4}-\lambda_{3}\right)\rho E^{*}\Rightarrow 2w_{3}u_{3}-\left(\lambda_{4}-\lambda_{3}\right)\rho E^{*}=0∴u_{3}^{*}=\frac{\left(\lambda_{4}-\lambda_{3}\right)\rho E^{*}}{2w_{3}},\\ u_{1}^{*}=\frac{\left(\lambda_{2}-\lambda_{1}\right)\gamma S^{*}+\lambda_{6}\theta V^{*}}{2w_{1}},\\ u_{2}^{*}=\frac{\left(\lambda_{4}-\lambda_{5}\right)\tau I^{*}+\left(\lambda_{6}-\lambda_{5}\right)\kappa R_{1}^{*}}{2w_{2}},\\ u_{1}^{*}=\frac{\left(\lambda_{4}-\lambda_{3}\right)\rho E^{*}}{2w_{3}}. \end{array}$$

**Theorem 7 .**

Given the optimal control vector (*u*_1_^∗^(*t*), *u*_2_^∗^(*t*), *u*_3_^∗^(*t*)) and the solutions *S*^∗^, *V*^∗^, *E*^∗^, *I*^∗^, *R*_1_^∗^, *R*^∗^ of the corresponding state system (34) and (35) that minimise the objective functional (*J*) over ∪, then there exist adjoint variables *λ*_1_, *λ*_2_, *λ*_3_, *λ*_4_, *λ*_5_, and *λ*_6_, where

(73) $$\begin{array}{c} u_{1}^{*}\left(t\right)=\max\left\{0,\min\left(1,\frac{\left(\lambda_{2}-\lambda_{1}\right)\gamma S^{*}+\lambda_{6}\theta V^{*}}{2w_{1}}\right)\right\},\\ u_{2}^{*}\left(t\right)=\max\left\{0,\min\left(1,\frac{\left(\lambda_{4}-\lambda_{5}\right)\tau I^{*}+\left(\lambda_{6}-\lambda_{5}\right)\kappa R_{1}^{*}}{2w_{2}}\right)\right\},\\ u_{3}^{*}\left(t\right)=\max\left\{0,\min\left(1,\frac{\left(\lambda_{4}-\lambda_{3}\right)\rho E^{*}}{2w_{3}}\right)\right\}, \end{array}$$

where *λ*_1_, *λ*_2_, *λ*_3_, *λ*_4_, *λ*_5_, and *λ*_6_ are the solutions of equations (28) and (30).

**Proof**

The presence of optimal control is as an aftereffect of the convexity of the integral of *J* regarding *u*_1_, *u*_2_, and *u*_3_, the Lipschitz property of the state system concerning the state factors from the earlier boundedness of the state arrangements [22, 23].

The differential conditions administering the adjoint factors are acquired by separation of the Hamiltonian work, assessed at the ideal control. By standard control contentions including the limits on the control, we conclude

(74) $$\begin{array}{c} \left.\begin{array}{c} u_{1}^{*}=\left\{\begin{array}{c} 0,\text{if }\eta_{1}^{*}\leq 0\\ \eta_{1}^{*},\text{if }0<\eta_{1}^{*}<1\\ 1,\text{if }\eta_{1}^{*}\geq 1 \end{array}\right.u_{2}^{*}=\left\{\begin{array}{c} 0,\text{if }\eta_{2}^{*}\leq 0\\ \eta_{2}^{*},\text{if }0<\eta_{2}^{*}<1\\ 1,\text{if }\eta_{2}^{*}\geq 1 \end{array}\right.u_{3}^{*}=\left\{\begin{array}{c} 0,\text{if }\eta_{3}^{*}\leq 0\\ \eta_{3}^{*},\text{if }0<\eta_{3}^{*}<1\\ 1,\text{if }\eta_{3}^{*}\geq 1 \end{array}\right. \end{array}\right\}, \end{array}$$

where *η*_1_^∗^ = ((*λ*_1_ − *λ*_2_)*γS*^∗^ + *λ*_6_*θV*^∗^)/2*w*_1_, *η*_2_^∗^ = ((*λ*_4_ − *λ*_5_)*τI*^∗^ + (*λ*_6_ − *λ*_5_)*κR*_1_^∗^)/2*w*_2_, and *η*_3_^∗^ = (*λ*_4_ − *λ*_3_)*ρE*^∗^/2*w*_3_.

## 5. Numerical Results

The state systems, adjoint equations, and the transversality terms are solved simultaneously to get the optimal strategies. The optimal problem is a two-point boundary value problem with two abstracted boundary conditions at initial times *t* = 0 and *t* = *t*_*f*_, where *t*_*f*_ = 3 months. This represents the period at which preventive strategies and treatment are expected to be stopped. The numerical simulation was conducted by solving the state equations, the adjoint equations, and the transversality conditions using the Runge-Kutta fourth-order scheme by guessing the controls over a simulated time. We then use the current iteration of the state equation, the adjoint equations, and the transversality conditions by a backward method. Further iterations are done until values of the unknown variables at the previous iteration are very close to those at the present iteration [18, 24, 25].

Table 3 shows the various parameter values used in the TB model simulations.

### 5.1. Strategy 1: Treatment, Prevention, and Vaccination of the Susceptible Population

Objective functional was optimised by using treatment, prevention, and vaccination as control measures. As a result of these control measures, there have been significant reduction of infections and an increase in the number of recovered populations as shown in Figures 2 and 3.

### 5.2. Strategy 2: Prevention and Treatment of the Infected Population

Objective functional was optimised by using prevention, vaccination, and treatment as control measures. The outcome of these control measures indicates a reduction of the population infected and increased recoveries, indicating that these variables have greatly impacted in the combat of the spread of infections as shown in Figures 4 and 5.

### 5.3. Strategy 3: Vaccination and Treatment of the Infected Population

Objective functional was optimised by using treatment, vaccination, and prevention of the susceptible population as control measures. Figures 6 and 7 show the effects of treatment and vaccination, respectively: an increase in the recovery population, a decrease in the infectious population, and a decrease in the number of population susceptible.

## 6. Conclusion

A deterministic model for tuberculosis was formulated and analysed. The basic reproductive number for the TB model is estimated using the next-generation matrix method.

The equilibrium points of the TB model and their local and global stability were determined. It was established that if the basic reproductive number was less than unity (*R*_0_ < 1), then the disease-free equilibrium is stable and unstable if R_0_ > 1. Furthermore, we investigated the optimal prevention, treatment, and vaccination as control measures for the disease.

Objective functional was optimised by using treatment, prevention, and vaccination as control measures. As a result of these control measures, there have been significant reduction of infections and an increase in the number of recovered populations as shown in Figures 2 and 3.

Objective functional was optimised by using prevention, vaccination, and treatment as control measures. The outcome of these control measures indicates a reduction of the population infected and increased recoveries as shown in Figures 4 and 5, indicating that these variables have greatly impacted in the combat of the spread of infections.

Objective functional was optimised by using treatment, vaccination, and prevention of the susceptible population as control measures. An increase in the recovery population, a decrease in the infectious population, and a decrease in the number of population susceptible are shown in Figures 6 and 7.

It was established that the best control measure in combating tuberculosis infections is prevention and vaccination of the susceptible population.

## Figures and Tables

**Figure 1:** Tuberculosis model flow diagram.

**Figure 2:** Optimal treatment of the infected population.

**Figure 3:** Optimal prevention and vaccination of the susceptible population.

**Figure 4:** Optimal prevention and treatment of the infected population.

**Figure 5:** Optimal prevention and vaccination of the susceptible population.

**Figure 6:** Optimal treatment of the population infected.

**Figure 7:** Optimal vaccination of the susceptible population.

**Table 1:** Variable description.

Variables	Description
*S*	Susceptible persons
*V*	Vaccinated persons
*E*	Exposed persons
*I*	TB-infected persons
*R*_1_	Individuals resistant to treatment
*R*	Recovered persons

**Table 2:** Parameter description.

Parameters	Description
*Λ*	Recruitment of susceptible individuals
*M*	Immigrants into the susceptible and infectious compartments
*α*	Rate of inflow of immigrants into the susceptible compartment
*σ*	Rate at which the cured lose their immunity
*μ*	Rate of natural mortality
*γ*	Rate of vaccination of susceptible individuals
*θ*	Rate at which the vaccinated recover
*β*	Rate at which the susceptible individuals are exposed to Mtb
*ρ*	Rate at which unprotected individuals get infected
*δ*	Disease-induced death rate
*κ*	Rate of recovery after treatment
*τ*	Rate of resistance to the treatment
(1 − *α*)	Rate of inflows of immigrants into the infected compartment

**Table 3:** Numerical values.

Parameter	Value	Reference
*Λ*	10	Assumed
*α*	0.9	[26]
*β*	0.05	Assumed
*γ*	0.2	Assumed
*σ*	0.4	Assumed
*μ*	0.01874	[27]
*θ*	0.1	Assumed
*ρ*	0.00114	[27]
*δ*	0.1577	[27]
*κ*	1.00	Assumed
*τ*	0.4	[28]

## Data Availability

Some of the parameter values are assumed, and others are taken from published articles and are cited in this paper. These published articles are also cited at relevant places within the text as references.
